The article "Effect of Cu Doping on ZnO Nanoparticles as a Photocatalyst for the Removal of Organic Wastewater" was retracted in 2023. Reasons: signs of a paper mill; compromised peer review; unreliable results or conclusions.

# Effect of Cu Doping on ZnO Nanoparticles as a Photocatalyst for the Removal of Organic Wastewater

**DOI:** 10.1155/2022/9459886

**Published:** 2022-06-30

**Authors:** Awais Khalid, Pervaiz Ahmad, Abdulhameed Khan, Saleh Muhammad, Mayeen Uddin Khandaker, Md. Mottahir Alam, Mohd Asim, Israf Ud Din, Ratiram G. Chaudhary, Dileep Kumar, Rohit Sharma, Mohammad Rashed Iqbal Faruque, Talha Bin Emran

**Affiliations:** ^1^Department of Physics, Hazara University Mansehra, Mansehra 21300, Khyber Pakhtunkhwa, Pakistan; ^2^Department of Physics, University of Azad Jammu and Kashmir, Muzaffarabad 13100, Pakistan; ^3^Department of Biotechnology, University of Azad Jammu and Kashmir, Muzaffarabad, Pakistan; ^4^Center for Applied Physics and Radiation Technologies, School of Engineering and Technology, Sunway University, Bandar Sunway 47500, Selangor, Malaysia; ^5^Department of Electrical and Computer Engineering, Faculty of Engineering, King Abdulaziz University, Jeddah 21589, Saudi Arabia; ^6^Department of Chemistry, Faculty of Science, University of Jeddah, Jeddah 21589, Saudi Arabia; ^7^Department of Chemistry, College of Science and Humanities, Prince Sattam Bin Abdulaziz University, P.O. Box 173, Al-Kharj 11942, Saudi Arabia; ^8^Post Graduate Department of Chemistry, Seth Kesarimal Porwal College of Arts, Commerce and Science, Kamptee 441001, India; ^9^Poona College of Pharmacy, Bharati Vidyapeeth (Deemed to Be) University, Pune, Maharashtra 411038, India; ^10^Department of Rasashastra and Bhaishajya Kalpana, Faculty of Ayurveda, Institute of Medical Sciences, Banaras Hindu University, Varanasi 221005, Uttar Pradesh, India; ^11^Space Science Center (ANGKASA), Universiti Kebangsaan Malaysia, 43600 UKM, Bangi, Selangor, Malaysia; ^12^Department of Pharmacy, BGC Trust University Bangladesh, Chittagong 4381, Bangladesh; ^13^Department of Pharmacy, Faculty of Allied Health Sciences, Daffodil International University, Dhaka 1207, Bangladesh

## Abstract

Environmental problems with chemical and biological water pollution have become a major concern for society. Providing people with safe and affordable water is a grand challenge of the 21st century. The study investigates the photocatalytic degradation capabilities of hydrothermally prepared pure and Cu-doped ZnO nanoparticles (NPs) for the elimination of dye pollutants. A simple, cost-effective hydrothermal process is employed to synthesize the Cu-doped ZnO NPs. The photocatalytic dye degradation activity of the synthesized Cu-doped ZnO NPs is tested by using methylene blue (MB) dye. In addition, the parameters that affect photodegradation efficiency, such as catalyst concentration, starting potential of hydrogen (pH), and dye concentration, were also assessed. The dye degradation is found to be directly proportional to the irradiation time, as 94% of the MB dye is degraded in 2 hrs. Similarly, the dye degradation shows an inverse relation to the MB dye concentration, as the degradation reduced from 94% to 20% when the MB concentration increases from 5 ppm to 80 ppm. The synthesized cost-effective and environmentally friendly Cu-doped ZnO NPs exhibit improved photocatalytic activity against MB dye and can therefore be employed in wastewater treatment materials.

The article "Effect of Cu Doping on ZnO Nanoparticles as a Photocatalyst for the Removal of Organic Wastewater" was retracted in 2023. Reasons: signs of a paper mill; compromised peer review; unreliable results or conclusions.

## 1. Introduction

Contaminated water from industries spilled into rivers after manufacturing a range of products in the sectors. Several chemical components present in this contaminated effluent may result in environmental issues. Chemical dye, organic and mineral materials, and synthetic dye all come from industrial, urban, and agricultural resources, with chemical dye being the maximum harmful pollutant emanating from fabric industries [1–3]. Many industries use water treatment plants to eliminate pollution from wastewater at a small price for environmental benefits [4–6]. This helps to improve and conserve the quality of water for drinking and other purposes. In the industrial sector, many treatments (recycling processes) are used to purify contaminated water. Heterogeneous photocatalysis is a frequent and simple approach. Heterogeneous photocatalytic treatment of organic pollutants in water is a promising alternative [7, 8]. The higher the defects or surface-to-volume ratio is, the more the photocatalytic effect of oxides is determined. In the ongoing process of photodegradation, transition metal (TM) oxides are used as catalysts [9]. Doping TM in oxides raises the crystal defect and modifies the optical band by changing the absorbance to a higher wavelength [10]. Zinc oxide (ZnO) is a potential photocatalytic material with a band gap of 3.4 eV [11, 12]. ZnO NPs are being investigated as a catalyst for the degradation of organic contaminants due to their high crystallinity, greater surface activity, and microstructural characteristics [13].

To improve the characteristics and usefulness of ZnO NPs at the nanoscale, various dopant materials, including transition metals (Mn, Fe, Cr, Co, and Cu), were required [1, 2, 14]. As a result of transition metals doping, the surfaces of these NPs are transformed to exhibit greater features such as a larger surface-to-volume ratio and compact size, allowing them to actively take part in photocatalysis and other applications. Cu^2+^ is reported to influence the structural, electrical, optical, biological, and magnetic aspects of the ZnO NPs more than any other dopants [15]. Cu^2+^ is the greatest alternative for biomedical applications because of its nontoxicity and its ionic radii that are comparable to those of Zn^2+^ (0.73 and 0.74) [16]. By incorporating Zn into a CuO crystal structure or Cu into a ZnO crystal structure, the combined dye degradation capabilities of ZnO and CuO can be explored [17]. Furthermore, the doping process results in greater electrical conductivity to the dopants. It can quickly adjust or modify the ZnO's physical and chemical properties. Likewise, Cu-doped ZnO NPs boost the storage capacity and energy conversion efficiency of electrochemical cells [16].

The article "Effect of Cu Doping on ZnO Nanoparticles as a Photocatalyst for the Removal of Organic Wastewater" was retracted in 2023. Reasons: signs of a paper mill; compromised peer review; unreliable results or conclusions.

Cu opted as a dopant material in ZnO to improve photocatalytic efficiency because it has influential luminous mediators by generating localized trapping tiers in the band gap to decrease recombination of charged carriers (photogenerated) [18]. It has physicochemical and microstructure features, the same as Zn [19]. Cu is used as a doping element for photocatalysis because of its unique features [20, 21]. The substitution of Cu ions in the ZnO lattice due to variations in the active mass and force in the native lattice also affects lattice dynamics, resulting in optical vibration modes at the Brillouin zone center. The occurrence of resident vibrational modes linked with external impurities and phase separation can be detected as a result of Cu ions doping [22].

Several approaches have been documented in the past due to the remarkable improvement in the characteristics of Cu-doped ZnO NPs. By using the coprecipitation technique, Cu-doped ZnO NPs are synthesized, which have a band gap equal to 3.4 eV. Copper concentration as a dopant was identified to play a significant role in improving photoluminescence characteristics [23]. The mechanically aided thermal breakdown technique also produced nanorods from pure and Cu-doped ZnO. Catalytic possessions of Cu-doped ZnO nanorods were discovered better than pure ZnO nanorods. To synthesize Cu-doped ZnO NPs, a variety of approaches have been reported, including coprecipitation, sol-gel, vapor transport technique, sol-gel combustion synthesis, and hydrothermal synthesis [24]. In the majority of the documented synthesis procedures, the Cu contents were reported to be insufficient to adjust the inherited characteristics of ZnO for the desired applications. Furthermore, almost all of the processes seemed complicated and time-consuming. In addition, in the final product, a few of the precursors were found as impurities. Unlike all of the preceding, a facile and feasible hydrothermal approach that is based on a precursor mixture of ZnCl_2_, CuCl_2_.2H_2_O, and NaOH has been investigated. The types of precursors, their concentrations, and the catalyst were also carefully selected with the ultimate product's composition in mind. The precursors can interact catalytically (after early breakdown) to create the bulk product (ZnO) in the presence of a Cu metallic catalyst. ZnO in bulk is converted to a smaller scale (nanometer) and doped with Cu by using copper's double-action (released from CuCl_2_.2H_2_O).

The article "Effect of Cu Doping on ZnO Nanoparticles as a Photocatalyst for the Removal of Organic Wastewater" was retracted in 2023. Reasons: signs of a paper mill; compromised peer review; unreliable results or conclusions.

A number of studies have been reported including Ag: ZnO/lignin [19], La: ZnO/metasystox [21], Co: ZnO and Mn: ZnO/methyl orange [20], Cu: ZnO/crystal violet [18], Fe: ZnO, Mg: ZnO, and Ca: ZnO/phenol [22], nitrogen-doped ZnO/bisphenol A under visible light irradiation [25], Nb: ZnO/methylene blue under UV irradiation [24], and Ag: ZnO/rhodamine B under UV and visible light irradiation [23]. The photocatalytic activity of ZnO was enhanced by doping in all these studies. It is worth mentioning that most of the investigations have not included photodegradation of methylene blue when exposed to UV light. The current work is unique in terms of precursors, dye, and experimental procedure in comparison with the published literature, as shown in Table 1.

Doping is the most widely researched strategy to modify nanoparticle (photocatalytic) characteristics. Furthermore, metal-doped ZnO NPs have been found to have maximum photocatalytic dye degradation abilities than pure ZnO NPs. The study aims to use a hydrothermal technique to synthesize Cu-doped ZnO NPs and investigate their photocatalytic abilities for the elimination of dye pollutants. In addition, the parameters that affect photodegradation efficiency, such as catalyst concentration, starting pH, and dye concentration, were assessed.

## 2. Materials and Methods

### 2.1. Preparation of Cu-Doped ZnO Nanoparticles

ZnCl_2_, CuCl_2_.2H_2_O, and NaOH were taken as precursors and procured from Sigma Aldrich. A mixture of ZnCl_2_ (1.5 g) is dissolved into deionized water (50 mL). After that, 1.2 g of NaOH is dissolved in 25 mL distilled water and poured into the homogenous solution of CuCl_2_.2H_2_O and ZnCl_2_ that has already been prepared. To prepare the doped sample, CuCl_2_.2H_2_O (0.25 g) and ZnCl_2_ (1.5 g) are dissolved into deionized water (50 mL) following the same procedure used for pure ZnO. After that, the solution is agitated for 30 minutes at room temperature. Consequently, several droplets of ethanol (10 ml) were poured into the solvent mixture. The solution is then taken into an autoclave (100 ml) and placed for 22 hours at 170°C in a hot air oven to react hydrothermally [8]. Finally, a white precipitate was obtained. Afterward, the white precipitate is washed with ethanol (2 times) followed by distilled water and then dried at 130 C for 1.5 hours in the oven.

The article "Effect of Cu Doping on ZnO Nanoparticles as a Photocatalyst for the Removal of Organic Wastewater" was retracted in 2023. Reasons: signs of a paper mill; compromised peer review; unreliable results or conclusions.

### 2.2. Characterization Tools

Field emission scanning electron microscopy (FE-SEM) was used to examine the shape and morphology of the Cu-doped ZnO NPs. X-ray photoelectron spectroscopy (XPS) and X-ray diffraction (XRD) were used to investigate the phase and crystal structure of the as-synthesized Cu-doped ZnO samples. A dispersive micro-Raman system with a 514 nm diode laser was used to record the sample's Raman spectra (in the range of 200–600 cm^−1^). Fluorescence spectrometer was used to investigate the absorption and photoluminescence of the powders.

### 2.3. Photocatalytic Activity of Cu-Doped ZnO NPs

Methylene blue (MB) dye (aqueous) was used to examine the photocatalytic degradation of Cu-doped ZnO NPs. The dye solution was irradiated by using a UV-C lamp from OSRAM. In the FL-PhR, four OSRAM UV-C lamps (*λ* = 254 nm) were employed. The power of each lamp was 8 watts, making the entire power 32 watts. Furthermore, 0.07 g of Cu-doped ZnO NPs was used as a catalyst in a 10 mL MB solution with a 5 ppm concentration (MB). The solutions were exposed to the UV light on a rotatory mover and shaker for 120 minutes (2 h) at room temperature. To remove the photocatalyst and evaluate the degrading effectiveness of MB, the reaction solutions were taken for absorption measurements by a UV-Vis (Systronics 2002) spectrophotometer after every 20 minutes.

## 3. Results and Discussion

Catalysts are used in a variety of approaches to synthesize bulk and nanomaterials as well as to dope (change or modify their properties). To prepare Cu-doped ZnO NPs, one such approach was proposed and implemented. CuCl_2_ is formed when NaOH catalyzes the reaction. The reaction between CuCl_2_.2H_2_O and ZnCl_2_ is permitted. As a result of the reaction, bulk ZnO and Cu were formed. Cu is also set to operate in two different methods. Cu first acts as a catalyst to reduce the size of ZnO NPs from bigger (bulk) to smaller (nano) and then regulates himself as a dopant in the ZnO lattice sites to generate ZnO doped with Cu.

### 3.1. X-Ray Diffraction (XRD) Analysis

Figure 1 shows the detected XRD pattern for pure and Cu-doped ZnO NPs. Structure, phase, and crystallite size of the samples were established by the peak's intensity and position. On the diffractogram, peaks 20 appear at 31.85°, 34.39°, 36.47°, 47.57°, 56.67°, 62.79°, 66.51°, 67.76°, 69.09°, 74.25°, and 75.83° corresponding to (100), (002), (101), (102), (110), (103), (200), (112), (201), (004), and (202) planes according to JCPDS card No. 89-7102 in pure and ZnO doped with Cu, respectively [25]. There are numerous other peaks on the radiograph, including 30.88°, 38.76°, and 53.47°, which are related to (100), (111), and (020) in Cu (II) oxide, while the peaks laying at 44.52° and 50.23° correspond to (111) and (200) planes in copper (FCC phase), respectively [36]. The appearance of CuO and Cu in the as-synthesized ZnO confirms Cu doping. The crystallite size of pure ZnO and Cu-doped ZnO samples was calculated using Scherrer's formula. The crystallite size was initially 45 nm which reduced to 34 nm on copper doping.

The article "Effect of Cu Doping on ZnO Nanoparticles as a Photocatalyst for the Removal of Organic Wastewater" was retracted in 2023. Reasons: signs of a paper mill; compromised peer review; unreliable results or conclusions.

### 3.2. Field Emission Scanning Electron Microscope (FE-SEM) Analysis

FE-SEM is used to observe the apparent morphology of hydrothermally synthesized ZnO and Cu-doped ZnO NPs.  Figure 2 shows the FE-SEM micrographs of the as-synthesized pure ZnO and Cu-doped ZnO NPs. In both Figures 2(a) and 2(b) micrographs, pure ZnO appears to have the morphology of nanosheets that have been trimmed by the inclusion of Cu. At the bottom, most of the Cu-doped ZnO NPs appear to be small discrete cotton packs stacked on top of each other. As observed in Figure 2(c), the majority of the smaller particles are tightly packed alongside others at the bottom.  Figure 2(d) demonstrates that the solid particles are agglomerated and positioned at the top. The agglomerated packets appear to represent the prepared bulk ZnO generated by the precursor's initial reactions and made up of multiple nanosized particles. The catalytic reaction of Cu may have brought these particles to the nanoscale. The Cu component affects the size and morphology of ZnO NPs. These findings are in close agreement with the available literature [37].

### 3.3. X-Ray Photoelectron Spectroscopy (XPS) Analysis

The bonding characteristics, valence states, and chemical compositions of the as-produced Cu-doped ZnO NPs reported in the X-ray photoelectron spectroscopy (XPS) are shown in Figure 3. Cu 2p peaks, Zn 2p peaks, and O 1s peak were found in the XPS study. The sample contains almost no magnetic impurities or precursor materials. Furthermore, a 285 eV C 1s signal is identified, which could be attributable to hydrocarbon contamination (this could be because the material was exposed to the air before being characterized).  Figure 3(a) shows the XPS survey with the spots labeled with the respective elements' binding energies. The survey reveals the high intensities of Cu 2p peaks (Cu contents) along with Zn 2p and O 1s peaks. Two prominent peaks can be seen in Figure 3(b), which belong to the spin-orbit of Zn 2p_3/2_ and Zn 2p_1/2_ at binding energies of 1022.1 and 1045.2 eV, accordingly. There is no noticeable peak shift, and the values are identical to those found in a ZnO (pure) sample. This indicates that, in the ZnO lattice, Zn exists in its +2-oxidation state. The high-resolution Gaussian-fitted XPS scans are shown in Figure 3(c). At 934.1 and 954.3 eV (binding energies), the Cu core level divides into Cu 2p_1/2_ and Cu 2p_3/2_. These findings support the idea that Cu seems to have a bivalent valence state [38]. Cupric oxide (Cu^2+^) is also linked to the satellite peak observed in the 940–945 eV range [39]. This shows that Cu ions (Cu^2+^) were oxidized in ZnO NPs and replaced at the Zn^2+^ position in the ZnO crystal. The enlarged O 1s peak is shown in Figure 3(d). In ZnO (wurtzite structure), the large peak in Zn-O bonding is attributed to O^2−^ ions with a binding energy of 530.9 eV. O^2–^ and O^–^ ions in oxygen lacking portions of the sample matrix are responsible for the twisted peak at 532.6 eV [40].

The article "Effect of Cu Doping on ZnO Nanoparticles as a Photocatalyst for the Removal of Organic Wastewater" was retracted in 2023. Reasons: signs of a paper mill; compromised peer review; unreliable results or conclusions.

### 3.4. Raman Spectroscopic Analysis

Raman spectroscopic studies were carried out in the 200–600 nm range. The observed Raman spectra in Figure 4 exhibit peaks at 355, 434, and 493 cm^−1^ for ZnO and Cu-doped ZnO NPs, accordingly. The E2 (high), E2H-E2L, transverse optical (TO), and A1 modes are responsible for these peaks [41]. Based on the literature, when the Cu doping content rises, the peak intensity in the spectra decreases, and the A1 (TO) phonon mode disappears. Additional Raman spectra peaks have been attributed to other optical modes, according to group theory. The polarized A1 and E1 modes can be separated into longitudinal optical (LO) and transverse optical (TO) phonons [42].

### 3.5. Photoluminescence Spectroscopy (PL) Analysis

Photoluminescence spectroscopy (PL) is used to examine the optical properties of the as-prepared materials, such as the influence of Cu on ZnO.  Figure 5 depicts the PL spectra of all the as-produced materials. There are two emission bands in the spectra. The spectrum of undoped ZnO comprises two peaks: one in the weak (UV) range, which corresponds to near band edge emission, and the second in the strong (visible) range. Exciton-related transitions were responsible for the weak region, while crystal defects such as oxygen and Zn vacancies were responsible for strong visible emission [43]. Cu has been confirmed to have a valence state of +2 in ZnO. Under the 325 nm excitation wavelength, the photoluminescence intensity dropped as the Cu doping concentration incorporated. The PL spectra were visible in all produced samples in UV and Vis range. At roughly 37°C, faint UV bands were shown for both pure and Cu-doped ZnO NPs. In the UV and Vis range, PL spectra were visible in all of the obtained samples. Weak UV bands were found at around 377, 381, 380, and 392 nm in pure ZnO and Cu-doped ZnO, which corresponded to near band gap excitonic emission. For pure and Cu-doped ZnO, the electronic transition in the band gap between the defect levels generates strong emission bands in the visible range at 535 nm, 547 nm, 556 nm, and 569 nm. PL spectra can thus be used to examine both the band gap and the relative energy positions of subband gap defect states. The green emission at 569 nm is caused by oxygen vacancies [44]. The UV and Vis bands were indistinguishable because the PL spectra were broad.

The article "Effect of Cu Doping on ZnO Nanoparticles as a Photocatalyst for the Removal of Organic Wastewater" was retracted in 2023. Reasons: signs of a paper mill; compromised peer review; unreliable results or conclusions.

### 3.6. Diffuse Reflectance Spectroscopy (DRS) Analysis

DRS is a versatile method that allows us to properly quantify the flux per wavelength of light rebounded from a sample in a scattered way. When incoming radiation illuminates powdered samples, the result is diffuse lighting. The room temperature reflectance spectra of the produced nanostructures are shown in Figure 6. The band gap value and reflectance of pure and Cu-doped ZnO NPs were calculated by using DRS spectra. The Kubelka–Munk function *F* (*R*) can be used to calculate the sample's diffuse reflectance (*R*). As in Figure 6, by introducing Cu content, the absorption boundary could move toward lower wavelengths. The quantum confinement phenomena could be responsible for the blue shift [45].

### 3.7. UV-Vis Spectroscopy Analysis

Figure 7 shows the observed UV-Vis absorption spectrum in the 300–700 nm range for synthesized samples of pure and Cu-doped ZnO NPs. In Figure 7(a), the absorbance of the pure ZnO sample seems to be lowest and increases with the addition of Cu content in ZnO. A variation in the wavelength of the peaks having maximum absorbance is seen in the UV-Vis spectra of pure and Cu-doped ZnO NPs. The band gap of the obtained ZnO and Cu-doped ZnO is shown in Figure 7(b). Initially, the band gap of the pure sample is measured as 3.17 eV and reduced to 3.06 eV for the Cu-doped ZnO sample.

### 3.8. Photocatalytic Degradation of MB by Cu-Doped ZnO Nanoparticles

Under ultraviolet (UV) light, the photocatalytic activity of the resulting pure and Cu-doped ZnO NPs was determined in comparison to the MB dye. For the MB dye degrading process, the typical absorption peak at 670 nm was employed as a reference.  Figure 8 shows the absorption spectra of an aqueous solution of MB in the presence of Cu-doped ZnO NPs for various time intervals (degradation versus time). The MB dye degradation (absorbance) is found to be inversely proportional to UV irradiation time. The characteristic strength of the MB peaks was observed to reduce with increasing exposure duration, as shown in Figure 8(a). This shows that the MB dye has degraded in the presence of nanoparticles. From Figure 8, an additional peak was observed with declining intensity at 612 nm. This demonstrates that the Cu atom has been doped into the ZnO structure.  Figure 8(b) shows the percent dye degradation at various time intervals. It was observed that, within 120 minutes, the amount of dye degraded was 94 ± 2%, demonstrating a steady rise in % degradation. Cu-doped ZnO is first photoexcited for the establishment of conduction band electrons and holes in the valence band, which is the suggested photodegradation pathway by Cu-doped ZnO for organic dye. A hole (+ive) is produced when an advanced e (electron) combines with water to form hydroxyl radicals. These radicals have been described as significant oxidizing agents that cause color fading [25]. Photogenerated electrons could potentially decrease dissolved oxygen, resulting in the formation of a superoxide anion radical. These anion radicals can also act as oxidizers, designed to destroy any absorbed organic molecules or compounds causing organic dye molecules to degrade near the catalyst's surface [46]. The rate of degradation calculated using the pseudo-first-order kinetics and schematic illustration for charge transportation process of Cu-doped ZnO NPs is shown in Figures 9(a) and 9(b).

The article "Effect of Cu Doping on ZnO Nanoparticles as a Photocatalyst for the Removal of Organic Wastewater" was retracted in 2023. Reasons: signs of a paper mill; compromised peer review; unreliable results or conclusions.

Dyes with various pH levels can be found in textile wastewater. As a result, investigating the role of pH in dye degradation is crucial. The charge on the catalyst, the position of the valence, and the conduction bands, as well as the formation of hydroxyl radicals, the characteristics of textile wastes, and the size of the catalyst, are all affected by pH [47, 48]. Cu-doped ZnO was investigated for 120 minutes at different pH (4, 6, 8, and 10) while keeping dye concentration constant (5 ppm). The pH of the solution was controlled using HNO_3_ and NaOH. The influence of pH on MB degradation is presented in Figure 10, indicating that there is a definite link between dye degradation and pH of the solution. According to the findings, almost 65% of the dye decomposed at pH 4. The MB degradation rate increases as the pH of the solution rises, reaching 80%, 85%, and 90%, respectively, for pH values 6, 8, and 10. The formation of hydroxyl radicals may be responsible for the significant degradation of MB dye. Furthermore, it was previously discovered that when employing ZnO and TiO_2_ as photocatalysts, the degradation of Reactive Orange 4 and Reactive Black 5 dye amplified with rising pH [49].

The effect of the quantity of catalyst has also been evaluated by using multiple catalyst concentrations (0.01 g, 0.02 g, 0.05 g, and 0.07 g). Absorption spectra of MB in aqueous solution by using various concentrations of catalyst (Cu-doped ZnO) before and after degradation are shown in Figure 11(a). The photodegradation of MB accelerates with the enhancement in the concentration of catalyst, as seen in the spectra. The improvement in degradation due to an increase in catalyst quantity could be associated with the increase in active sites. The quantity of superoxide and hydroxyl radicals increases, resulting in dye degradation. Percent (%) degradation of MB dye by using various concentrations of catalyst is shown in Figure 11(b), which shows that 0.01 g, 0.02 g, 0.05 g, and 0.07 g Cu-doped ZnO NPs (catalyst) degraded 30%, 50%, 75%, and 85% in 120 minutes (2 h). The variation in photodegradation was also observed due to variation in dye (MB) concentration. Various amounts of MB (5, 10, 25, 50, and 80 ppm) were used with decomposition rates of 94%, 80%, 65%, 35%, and 20%, respectively, by using a fixed amount of catalyst (0.05 g). As the content of MB increases, the rate of degradation reduces, as shown in Figure 12. This could be due to dye molecules absorbing UV light instead of catalyst molecules on the surface of the catalyst (Cu-doped ZnO). By blocking the active sites of photocatalysts with dye molecules, it contributes to the reduction of hydroxyl radicals [50]. Cu-doped ZnO NPs have the potential to be used in air and wastewater treatment resources based on their better catalytic activity in terms of time, pH, catalyst concentration, and dye concentration [48, 51–53].

The article "Effect of Cu Doping on ZnO Nanoparticles as a Photocatalyst for the Removal of Organic Wastewater" was retracted in 2023. Reasons: signs of a paper mill; compromised peer review; unreliable results or conclusions.

## 4. Conclusions

Cu-doped ZnO nanoparticles were prepared by using a hydrothermal method. State-of-the-art techniques XRD, FE-SEM, RAMAN, XPS, PL, DRS, and UV-Vis spectroscopy were used to study the morphology, structure, material composition, band gap, and dye degradation potential of Cu-doped ZnO nanoparticles. The liberated copper is considered to have a key role in the reduction in the size of pure and Cu-doped ZnO during the process. The findings indicate that 90 percent of the MB (dye) was degraded in 120 minutes, with 65%, 80%, 85%, and 90% degradation at pH 4, 6, 8, and 10. It seems that an alkaline condition is favorable for quick photodegradation of MB. As per the catalyst concentration analysis, 0.01 g of catalyst (Cu-doped ZnO) decomposed 30% of the dye, increasing to 85 percent with 0.07 g. The enhanced degradation with an increase in catalyst quantity could be due to the additional active sites. As a result, the amount of hydroxyl radicals and superoxide rises, causing dye degradation. Cu-doped ZnO NPs exhibit improved photocatalytic activity against MB dye. It is cost-effective and environmentally safe and can be employed in wastewater treatment materials.

## Figures and Tables

**Figure 1:** XRD pattern of pure and Cu-doped ZnO NPs demonstrating peaks for various components in the material.

The article "Effect of Cu Doping on ZnO Nanoparticles as a Photocatalyst for the Removal of Organic Wastewater" was retracted in 2023. Reasons: signs of a paper mill; compromised peer review; unreliable results or conclusions.

**Figure 2:** Undoped and Cu-doped ZnO FE-SEM micrographs: (a) low and (b) high magnifications of pure ZnO and (c) low and (d) high magnifications of Cu-doped ZnO NPs.

**Figure 3:** (a) XPS survey of Cu-doped ZnO NPs, (b) Zn 2p peaks (high resolution), (c) Cu 2p peaks (high resolution), and (d) O 1s peak.

**Figure 4:** Raman spectroscopic study of undoped and Cu-doped ZnO NPs.

**Figure 5:** PL spectra of pure and Cu-doped ZnO NPs.

**Figure 6:** DRS spectra of pure and Cu-doped ZnO NPs.

**Figure 7:** (a) UV-Vis absorption spectrum in the 300–700  nm range for synthesized samples of pure and Cu-doped ZnO NPs. (b) The band gap of the as-obtained ZnO and Cu-doped ZnO.

**Figure 8:** (a) Absorption spectrum of photodegraded MB by Cu-doped ZnO and (b) % degradation of methylene blue at various time intervals.

**Figure 9:** (a) Plot of ln (Co/Ct) versus time for illustrating the kinetics of photodegradation. (b) Charge transportation process of Cu-doped ZnO NPs leading to photocatalytic dye degradation.

**Figure 10:** Effect of pH on methylene blue degradation.

**Figure 11:** (a) Absorption spectra of MB dye by various concentrations of Cu-doped ZnO and (b) % degradation of methylene blue at various catalyst amounts.

**Figure 12:** Effect of MB concentration on degradation (%).

**Table 1:** Comparison of various parameters of Cu-doped ZnO NPs with published articles.

S. no/reference	Precursors	Temperature/time	Technique	Morphology	Product	Dye	Year
[25]	Zn (CH_3_COO)_2_ 2H_2_O and CuSO_4_ 5H_2_O	25 C/3 h	Sol-gel method	Nanoparticles	Cu-doped ZnO	Methyl orange	2011
[26]	ZnCl_2_ and CuCl_2_·5H_2_O	120 C/1 h	Coprecipitation method	Nanoparticles	Cu-doped ZnO	—	2014
[27]	Zn (NO_3_)_2_ 6H_2_O and CuSO_4_ 5H_2_O		Coprecipitation method	Nanoparticles	Cu-doped ZnO	Methylene blue	2015
[28]	Zn (NO_3_)_2_.6H_2_O and CuSO_4_ 5H_2_O	85 C/1 h	Hydrolysis and oxidizing process	Nanoparticles	Cu-doped ZnO	Benzylic alcohols	2015
[29]	Zn (CH_3_COO)_2_ 2H_2_O and CuCl_2_	450 C/5 h	Coprecipitation method	Nanoflakes	Cu-doped ZnO	3-styryl-chromones	2016
[30]	ZnSO_4_ and CuSO_4_	250 rpm/12 h	Soft chemical method	Nanoparticles	Cu-doped ZnO	Methylene blue	2017
[31]	Zn (NO_3_)_2_.6H_2_O and Cu (NO_3_)_2_	200 C/2 h	Green chemistry	Nanoparticles	Cu-doped ZnO	Acid black 234	2017
[32]	ZnCl_2_ and CuCl_2_	80 C/18 h	Coprecipitation method	Nanorods	Cu-doped ZnO	Diazinon	2017
[33]	Zn (NO_3_)_2_.6H_2_O and Cu (NO_3_)_2_	80 C/3 h	Coprecipitation method	Nanoparticles	Cu-doped ZnO	—	2019
[34]	Zn (CH_3_COO)_2_ 2H_2_O and Cu (CH_3_COO)_2_ 2H_2_O	100 C/2 h	Coprecipitation method	Nanoparticles	Cu-doped ZnO	Arsenic	2020
[35]	Zn (NO_3_)_2_ 6H_2_O and Cu (NO_3_)_2_ 5H_2_O	550 C/3 h	Flash combustion method	Nanoparticles	Cu-doped ZnO	Methyl green	2020
Our article	ZnCl_2_ and CuCl_2_.2H_2_O	170 C/22 h	Hydrothermal method	Nanoparticles	Cu-doped ZnO	Methylene blue	2021

The article "Effect of Cu Doping on ZnO Nanoparticles as a Photocatalyst for the Removal of Organic Wastewater" was retracted in 2023. Reasons: signs of a paper mill; compromised peer review; unreliable results or conclusions.

## Data Availability

The data used to support the findings of this study are included within the article.
